# Acute Kidney Injury in Patients with Liver Cirrhosis: Prevalence, Predictors, and In-Hospital Mortality at a District Hospital in Ghana

**DOI:** 10.1155/2022/4589767

**Published:** 2022-02-21

**Authors:** Amoako Duah, Francisca Duah, Daniel Ampofo-Boobi, Bright Peprah Addo, Foster Osei-Poku, Adwoa Agyei-Nkansah

**Affiliations:** ^1^Department of Medicine, University of Ghana Medical Centre, Accra, Ghana; ^2^Laboratory Department, Ga-North Municipal Hospital, Ofankor, Ghana; ^3^Department of Medicine, St. Dominic Hospital, Akwatia, Ghana; ^4^Department of Biostatistics, St. Dominic Hospital, Akwatia, Ghana; ^5^Department of Medicine, University of Ghana Medical School, Korle-Bu Teaching Hospital, Accra, Ghana

## Abstract

**Background:**

Acute kidney injury (AKI) is one of the most severe complications of cirrhosis and portends an ominous prognosis with an estimated mortality of about 50% in a month and 65% within a year. Infection and hypovolemia have been found to be the main precipitating factors of AKI in liver cirrhosis. Early detection and treatment of AKI may improve outcomes. AKI in patients with liver cirrhosis in Ghana and their impact on inpatient mortality are largely unknown. This study was aimed at determining the prevalence, precipitating factors, predictors, and in-hospital mortality of AKI in patients with liver cirrhosis admitted to a district hospital in Ghana.

**Methods:**

Consecutive hospitalized patients with liver cirrhosis from 1 January 2018 to 30 April 2020 were recruited. Patient's demographic data and clinical features were collected using a standardized questionnaire. Biochemical and haematological tests as well as abdominal ultrasound scans were done for all patients. All patients were then followed up until discharge or death.

**Results:**

There were 117 (65.4%) males out of the 179 patients with a mean age of 49.94 and 45.84 years for those with and without AKI, respectively. The prevalence of AKI was 27.9% (50/179). Out of 50 participants with AKI, 64.0% (32/50) died, contributing 41.0% of all in-patient mortality amongst participants. There was a significant association between AKI and death (*p* ≤ 0.001). The major precipitating factors of AKI were infections (60.0%), hypovolemia (20.0%) due to gastrointestinal bleeding and gastroenteritis, and refractory ascites (16.0%). Alkaline phosphatase, INR, model for end-stage liver disease sodium, sodium, and blood urea nitrogen were independent predictors of AKI.

**Conclusion:**

AKI was common among patients with liver cirrhosis with high in-patient mortality. Identification of these precipitants and independent predictors of AKI may lead to prompt and targeted treatment with reduction in patient mortality.

## 1. Introduction

Liver cirrhosis is a worrying medical condition globally, particularly in Ghana where hepatitis B and alcohol are important risk factors [1]. It is a sequel of all chronic liver diseases characterized by replacement of liver tissue by fibrosis, scar tissue, and regenerative nodules, resulting in increased loss of liver function [2]. Cirrhosis can remain compensated for many years before the development of a decompensating events. Decompensated cirrhosis is marked by the development of any of the following complications: jaundice, variceal hemorrhage, ascites, and encephalopathy. One of the deadly and common complications of liver cirrhosis, especially in decompensated cirrhosis, is AKI [3]. In patients with liver cirrhosis admitted to the hospital, 20% to 50% of them are diagnosed with acute kidney failure, while chronic kidney disease is present in approximately 1% [4–6]. AKI is one of the key predictors for short-term mortality in patients with liver cirrhosis with mortality rates as high as 90% [7, 8]. There is a remarkable increase in length of hospital stay with high financial burden on patients with AKI [9]. In decompensated liver cirrhosis patients, Child-Pugh score and its components, which have been generally used to assess the severity of hepatic dysfunction together with AKI, have been found to be strong predictors of death [3].

Formerly, AKI in cirrhosis was defined as a 50% increase in serum creatinine (SCr) with a final value above 133 *μ*mol/l [10]. Due to the high incidence of malnutrition and sarcopenia in patients with liver cirrhosis [11], this means milder degrees of AKI are not being diagnosed and therefore not given immediate attention and care. AKI is now defined as a rise in serum creatinine (SCr) of ≥50% from baseline or a rise in SCr by ≥26.5 *μ*mol/l in <48 h or equal to 1.5 times baseline, which has occurred within the prior 7 days [12, 13]. Hepatorenal syndrome (HRS) type 1 is a unique type of AKI.

Aetiology of AKI can be categorized into three main types. These are prerenal (results from decreased renal perfusion), intrinsic renal (acute tubular necrosis), and postrenal AKI. In patients on admission, acute tubular necrosis is a common type of intrinsic AKI. Prolonged hypotension leading to ischemia or nephrotoxic agents that are toxic to the tubular cells are the major causes of acute tubular necrosis. Enlargement of the prostate gland causing obstruction of the urinary tract is the common cause of postrenal AKI [2, 14]. The development of portal hypertension in patients with liver cirrhosis leading to a reduction in systemic vascular resistance as a result of primary arterial vasodilation in the splanchnic circulation is the primary cause of AKI in cirrhotics [15]. This mechanism primarily leads to hepatorenal syndrome. In addition, the underlying causes of liver cirrhosis can be the cause of intrinsic renal disease. These forms of nephropathy include glomerulonephritis associated with alcoholic cirrhosis and infections such as chronic hepatitis B and C and schistosomiasis [16]. Bacterial infections and hypovolemia resulting from gastrointestinal bleeding and over diuresis are other common causes of AKI [17].

Early identification and management of AKI may improve outcomes [18]. AKI in patients with liver cirrhosis in Ghana and their impact on inpatient mortality are largely unknown. This study was aimed at determining the prevalence, precipitating factors, predictors, and in-hospital mortality of AKI in patients with liver cirrhosis admitted at St. Dominic Hospital, Akwatia in Ghana.

## 2. Methods

### 2.1. Study Design, Site, and Participants

The research design was a prospective hospital-based study, conducted at the internal medicine department, St. Dominic hospital (SDH), Akwatia, from 1 January 2018 to 30th April 2020. The SDH is a 339-bedded mission hospital that serves Denkyembour district in the Eastern region of Ghana and serves as the main referral center for other district hospitals within the eastern region. The hospital provides various medical and surgical services including gastroenterology, neurology, general internal medicine, obstetrics and gynecology, child health, ophthalmology, general surgery, and endoscopy.

Liver transplantation services are not currently available at the study site and in Ghana as a whole. There is lack of local clinical expertise and inadequate infrastructure to support liver transplant in Ghana. Appropriate legal framework of organ transplantation and guidelines are also not available in Ghana. Presently, patients requiring liver transplants and can afford travel to foreign countries where the services are available to have it done.

Overall, one hundred and seventy-nine (179) patients with liver cirrhosis admitted to the medical wards of SDH were recruited over the study period. The sample size was determined using the Cochran formula for sample size calculation, with an estimated prevalence of 12.9% for liver cirrhosis worldwide [3] and a *Z*-score of 95% confidence interval level (1.96) and a level of significance of 0.05. The minimum sample size was calculated to be 171. Due to the high attrition rate for prospective studies, 179 participants were consecutively recruited after meeting study criteria and giving informed consent.

#### 2.1.1. Inclusion Criteria

1. All adult patients above 18 years with diagnosis of liver cirrhosis
2. Patients who provided informed consent

#### 2.1.2. Exclusion criteria

1. Patients with known preexisting chronic kidney disease
2. Patients who had undergone renal transplantation
3. Refusal to give informed consent

Diagnosis of liver cirrhosis was based on the presence of two or all three of the following [19]:

1. Clinical signs of chronic liver disease (clubbing, palmar erythema, spider naevi, gynaecomastia, distended abdominal veins, female pubic hair pattern, encephalopathy, splenomegaly, or ascites)
2. Impaired liver function consistent with cirrhosis (elevated INR and low serum albumin)
3. Ultrasound diagnosis of cirrhosis (Shrunken or enlarged nodular liver with increased echotexture, blunt edge, and distorted architecture, with or without a dilated portal vein, thickened gallbladder wall, splenomegaly, or ascites)

AKI in patients with liver cirrhosis was defined by any one of the following: a rise in serum creatinine (sCr) of ≥50% from baseline or a rise in sCr by ≥26.5 *μ*mol/l in <48 h, or a rise in sCr to ≥1.5 times baseline, occurring within the prior 7 days [13, 20]. Baseline creatinine values were taken from the three-month preadmission periods. Admission values were used if they were normal or if prehospitalization baselines were not available. Those with no prehospitalization creatinine values, sCr ≥ 133umol/l, were considered as having AKI at the time of admission. The staging of AKI in this study was adopted from a study published by Xu et al. [21]. AKI stage 1 was defined as a rise in sCr ≥ 26.5 *μ*mol/l or ≥1.5 to 2-fold from baseline, including AKI stages 1A (sCr ≥ 133 *μ*mol/l) and 1B (sCr ≥ 133 *μ*mol/l); AKI stage 2 was defined as a rise in sCr ≥ 2 to 3-fold from baseline; AKI stage 3 was defined as a rise in sCr ≥ 3-fold from baseline or sCr ≥ 353.6 *μ*mol/l with an acute increase in sCr ≥ 26.5 *μ*mol/l or initiation of renal replacement therapy. Initial AKI stage was defined as the stage of AKI first diagnosed during hospitalization. Progression of stage of AKI or no progression was determined by the last AKI stage close to discharge or death in relation to the initial AKI stage.

Patients with AKI associated with acute on chronic liver failure (ACLF) were differentiated from those with AKI and without ACLF.

In this study, ACLF was defined as acute worsening of preexisting liver cirrhosis (decompensated or compensated) usually related to a precipitating event and associated with short-term mortality due to multiple organ failure. Organ failure was defined using Chronic Liver Failure-Sequential Organ Failure (CLIF-SOFA) score which includes six types of organ failure: liver, renal, coagulation, cerebral, respiratory, and circulatory [22].

### 2.2. Data Collection

Appropriate questionnaires were administered to those who met the inclusion criteria and gave their consent to be part of the study after thoroughly explaining the study to them. The data collected included sociodemographic data (age, sex, occupation, etc.), clinical features (spider angioma, jaundice, abdominal pain, weight loss, confusion, hematemesis, palmar erythema, ascites, asterixis, hepatomegaly, splenomegaly, abdominal vein collaterals, etc.), and alcohol use. Initial data on laboratory and imaging findings were obtained within a day of admission. Ascites was graded as mild (detectable only on ultrasound), moderate (visible, moderate symmetrical abdominal distension), or severe (marked abdominal distension) [23]. Hepatic encephalopathy was graded from grade 0 to IV, as per the West Haven criteria [24]. Mean arterial pressure (MAP), partial pressure of arterial oxygen (PaO2), and pulse oximetric saturation (SpO2) were obtained.

Risk factors/aetiological spectrums of liver cirrhosis were defined as follows:

  Chronic HBV was defined as a positive HBsAg result
  Chronic HCV was defined as a positive anti-HCV antibody result

Alcoholic aetiology was made when patient's declared alcohol consumption was more than 21 units of alcohol for men or 14 units for women per week when measurable or local alcohol beverage consumption was three times per week in the past five years and correlated with biological abnormalities related to alcohol consumption [25].

Hepatic schistosomiasis was defined as the presence of Schistosoma mansoni ova in stool and/or ultrasound findings of hepatic schistosomiasis features such as periportal fibrosis.

NAFLD aetiology was made when patients have risk factors for NAFLD and its progression and excluding other causes of liver cirrhosis.

Unidentified aetiology refers to CLD patients in whom no etiology was traced.

### 2.3. Measurements

#### 2.3.1. Blood and Urine Tests

Ten (10) mls of blood was taken for hematological, biochemical, and serological tests. Hematological and biochemical workup included hemoglobin, total leukocyte count, platelet count, prothrombin time/INR, and serum concentrations of bilirubin (total and conjugated), protein, albumin, alanine aminotransferase (ALT), and aspartate aminotransferase (AST). Serum sodium, potassium, blood urea nitrogen (BUN), and creatinine were also done for all patients. All patients were tested for HBsAg and anti-HCV antibodies to determine the cause of liver cirrhosis. The Child-Pugh scoring (CPS) system was used for assessing the severity of liver disease on patient presentation (26). The scoring system takes into account the serum albumin, serum prothrombin time or international normalized ratio (INR), and bilirubin as well as the presence of fluid retention and encephalopathy; each of which is given a numerical score. There are 3 grades: A, B, and C depending on the total scores. Model for end-stage liver disease sodium (MELD-Na) was also calculated for all patients [24]. Urine analysis (proteins, leucocytes, erythrocytes, pus cell, and other urine abnormalities) was done for all patients. Those with a positive leucocyte or nitrite on urinalysis had a follow-up urine culture.

#### 2.3.2. Ascitic Fluid Analysis

Ascitic fluid analysis including cell count and differentials, albumin, and protein was done for all patients. Ascitic fluid culture: about 5-10 mls of ascitic fluid were collected during the diagnostic abdominal paracentesis and put into sterile culture bottle at the patient bed side. Ascitic fluid culture was done by an experienced biomedical scientist by inoculating the ascitic fluid onto the blood agar and MacConckey agar. The preliminary results were obtained after 48 hours, followed by conventional biochemical identification tests. The diagnosis of spontaneous bacterial peritonitis in patients with cirrhosis was based on the positive culture with no more than 1 species of organism and/or neutrophil cell counts in the ascitic fluid (>250/mm^3^) regardless of the result of the ascitic fluid culture.

#### 2.3.3. Imaging Studies

Abdominal ultrasound scan was conducted for all patients, and the following information was recorded: liver and spleen size, changes on the liver surface and edges, presence of ascites, kidney size, and presence of liver mass. In patients with clinical diagnosis of pneumonia, chest X-ray was done for all of them, and areas of consolidation were noted.

#### 2.3.4. Ethical Approval and Informed Consent

This study was conducted in accordance with the Helsinki Declaration on Human Experimentation, Sixth Revision (October 2008) and approved by the Institutional Ethical and Review Committee of the St. Dominic Hospital. The study was fully explained to the patients, and those who agreed to be part were asked to sign an informed consent. For patients who were drowsy, confused, and comatose on account of HE, written consent was obtained from caregivers.

#### 2.3.5. Statistical Analysis

Statistical Package for Social Sciences (IBM SPSS, version 23) statistical software was used to analyze the data. Descriptive statistics were undertaken for all variables and data presented in appropriate tables. A subgroup analysis was done to compare sociodemographic characteristics and clinical features of patients with AKI with and without ACLF. Etiology of cirrhosis of the liver and the prevalence of AKI were determined. Associations between AKI and the clinical or laboratory parameters using Chi-square were also determined. A multivariable regression analysis was conducted to determine if any of the clinical, laboratory parameters and prognostic scores (CPS, MELDNa) were a predictor of AKI. *p* value < 0.05 was considered statistically significant in all analysis.

## 3. Results

### 3.1. Demographic Characteristics and Clinical Features of Cirrhotic Patients with and without AKI

A total of 179 patients were recruited, comprising of 117 (65.4%) males. Their ages ranged from 20 to 77 years with a mean age of 49.94 and 45.84 years for those with and without AKI, respectively. The prevalence of AKI was 27.9% (50/179). Out of 50 participants with AKI, 64.0% (32/50) died, contributing to 41.0% of all inpatient mortality amongst participants. There was a strong association between AKI and death (*p* 0.001). The clinical features significantly associated with AKI were infection and encephalopathy. There was no difference in terms of duration of stay between patients admitted with and without AKI (*p* 0.578). Other demographics are as shown in Table 1.

### 3.2. Demographic Characteristics of Cirrhotic Patients with AKI with and without ACLF

In subgroup analyses, out of the 50 patients with AKI, ACLF was diagnosed in 16 patients with infection as the main precipitating factor. All the patients diagnosed with ACLF with AKI died compared with 47.1% of those with AKI without ACLF which was statistically significant (*p* 0.001) (Table 2).

### 3.3. Child-Pugh Classification

The majority of patients admitted had CPS class C, 64.8% (116/179), and class B, 26.3% (47/179) (Table 3).

### 3.4. Causes of Liver Cirrhosis

The major causes of liver cirrhosis were significant alcohol consumption and hepatitis B virus in 72 (40.2%) and 65 (36.3%) of participants, respectively. The other causes found were hepatitis C virus in 6 (3.4%), nonalcoholic fatty liver disease (NAFLD) in 5 (2.8%), and schistosomiasis in 4 (2.2%). In 13 (7.3%) of the patients, the causes of their liver cirrhosis were not identified, and other causes are as shown in Table 4.

### 3.5. Precipitating Factors for All AKI

The major precipitating factors of AKI were infections (30/50, 60.0%), hypovolemia (10/50, 20.0%) resulting from gastrointestinal bleeding (5/50, 10%) and gastroenteritis (5/50, 10%), and refractory ascites (8/50, 16.0%). Unknown precipitants accounted for 4.0% (2/50) (Table 5).

### 3.6. AKI Stage and Its Effect on In-Hospital Mortality

Out of the 50 patients diagnosed with AKI, the majority of them had AKI stages 2 and 3. Patients who died had 6 times the odds of having Stage 1b AKI (compared to those who had Stage 1a AKI though this was not statistically significant [COR (95%CI) = 6 (0.42–85.2)]. Stage 2 and 3 AKI was associated with increased odds (statistically significant) of mortality compared to stage 1a with odds ratios of 10.29 (1.02-103.95) and 48 (3.64-631.76), respectively (Table 6).

### 3.7. Laboratory Parameters of the Study Participants

The laboratory parameters associated with AKI were high bilirubin, mainly conjugated bilirubin, low serum albumin, high international normalize ratio (INR), low sodium and potassium, high creatinine and BUN, alkaline phosphatase (ALP), CPS, and MELDNa (Table 7).

### 3.8. Multivariable Regression Analysis of Independent Variables Associated with AKI

ALP, INR, MELDNa, sodium, and BUN were independent predictors of AKI (Table 8).

## 4. Discussion

AKI is one of the most severe and life-threatening complications of cirrhosis with an estimated mortality of about 50% in a month and 65% within a year [8]. Infection and hypovolemia mainly due to upper and lower gastrointestinal bleeding and over diuresis have been found to be the main precipitating factors of AKI in liver cirrhosis [16]. This study is aimed at determining the prevalence, precipitating factors, predictors, and in-hospital mortality of AKI in patients with liver cirrhosis admitted in a hospital in Ghana. This study represents the first ever report on AKI in patients with liver cirrhosis to the best of our knowledge in Ghana. The prevalence of AKI in this study was 27.9%, which is in agreement with the published literature [4, 5, 7]. A similar prevalence of 28.0% was reported by Gameiro et al. [26], in their study in Portugal. A lower prevalence of 12.9% and 17.0% were reported by Choi et al. [3] and Terra et al. [27], respectively, in their studies. Wu et al. [28] and Hampel et al. [29] also reported 23% and 25% of AKI in their patients, respectively, which were slightly lower than the prevalence obtained in this study. Lasheen et al. [2] and Lins et al. [30]reported a prevalence of 43.8% and 53.9% in their studies, respectively, which were higher than 27.9% in this current study. The difference maybe is a result of the demographic characteristics of the patients as well as the severity and etiology of liver disease, risk factors for AKI, and variations of several thresholds for serum creatinine used to define AKI.

Acute kidney failure can be triggered by events such as overdose of diuretics, gastrointestinal bleeding, large-volume paracentesis without albumin replacement, and bacterial infections [31]. The major precipitating factors in this study were infections (60.0%), hypovolemia due to UGIB and gastroenteritis (20.0%), and refractory ascites (16.0%). This is similar to the precipitating factors reported by Lasheen et al. [2] and Gomes et al. [32] in their study. They documented infection and hypovolemia as major precipitating factors of AKI. Belcher et al. [33] also published hypovolemia and infections as major precipitating factors. Triggers of AKI should be identified early and dealt on to improve the outcome of these patients.

The estimated mortality of patients with AKI in patients with liver cirrhosis is around 50% in a month and 65% within a year [8]. Belcher et al. [33] in a prospective multicentric study involving 192 cirrhotic patients reported 26% intrahospital mortality, while Scott et al. [34] reported intrahospital mortality of 31.8% in their study. Gomes et al. [32] and Allegretti et al. [35] documented mortality rates of 45% and 46% in their studies, respectively, within 3 months of AKI diagnosis. Wong et al. [36] also observed a 34% mortality rate in 30 days. Results of meta-analysis demonstrated that the overall mortality of renal dysfunction among patients with liver cirrhosis and UGIB was 46%, with significant heterogeneity [37]. In the current study, the mortality rate among patients with AKI was as high as 64.0%. However, in those admitted with AKI and concomitant ACLF, the mortality rate was 100%. This confirms the high short-term mortality associated with ACLF (22). Stages of AKI significantly influenced the in-hospital mortality in this study. Patients with more severe stages of AKI, i.e., stages 2 and 3, had the higher odds of mortality compared to those with stages 1A. This is similar to a study conducted by Xu et al. [21]. The variations among mortality rates maybe as a result of differences in the study populations, the underlying precipitating factors of AKI, etiology and severity of liver disease, stage of AKI, and resources available for managing the patients. Vasoactive drugs such as terlipressin have been found to improve the outcome of patients with liver cirrhosis and AKI, especially those precipitated by gastrointestinal bleeding [21]. None of the patients in this study was administered with terlipressin or any other vasoactive drugs because of nonavailability at the study site. Terlipressin and other vasoactive drugs are also not widely available in Ghana, are expensive, not covered by Ghana's national health insurance, and therefore are not affordable to the majority of patients. Patients with AKI in this study were managed by treating the precipitating factors and managing the underlying causes of liver cirrhosis.

Patients who developed AKI in this study had laboratory values suggesting more advanced liver disease: higher bilirubin and INR and lower albumin and sodium values. At the same time, CPS and MELDNa were higher in patients with AKI compared to those without. Patients with AKI had infection and encephalopathy more than those without. However, high BUN, high MELDNa, high INR, and ALP were clinical parameters and scores that were independent predictors of AKI. Tariq et al. [38] reported MELD, CPS stage C, presence of ascites, and presence of sepsis/septic shock as predictors associated with AKI. Gameiro et al. [39] in their study also identified MELDNa and neutrophil-to-lymphocyte ratio as an independent predictive factor of AKI. Other studies have also reported CPS, INR, total bilirubin, serum albumin, platelet count, MELD, total leucocyte count, SBP, and shock as risk factors for AKI [40]. Patients with advanced liver cirrhosis who develop infections should be screened early for AKI and treatment instituted to reduce mortality.

## 5. Conclusion

AKI was common among patients with liver cirrhosis admitted at SDH with high in-patient mortality especially AKI associated with ACLF. The major precipitating factors of AKI were infection, hypovolemia from gastrointestinal bleeding and gastroenteritis, and refractory ascites. ALP, INR, MELDNa, serum sodium, and BUN were independent predictors of AKI. Strategies to prevent and treat precipitating factors early may lead to an improvement in the outcome of these patients. A similar study should be done on a larger scale country-wide in multiple centres and regions to get a well-balanced prevalence of AKI. In addition, a study should be conducted to determine the prevalence of multidrug-resistant bacteria in these patients, which is increasing worldwide.

## Figures and Tables

**Table 1:** Demographic characteristics and clinical features of cirrhotic patients with and without AKI.

Demography	AKI, present (*N* = 50)	AKI, absent (*N* = 129)	*p* value
Age of patient (years, IQR)	49.94 (36.47, 63.47)	45.84 (33.05, 58.63)	0.6
*Sex of patient*			0.38
Male	30 (25.6)	87 (74.4)	
Female	20 (32.3)	42 (67.7)	
*Blood pressure (mmHg, IQR)*			
Systolic BP	106 (92.15, 119.85)	108.7 (93.8, 123.56)	0.268
Diastolic BP	68.52 (58.52, 78.52)	69.15 (58.86, 79.4)	0.713
Length of stay (days)	10.06 (2.69, 17.43)	10.67 (3.97, 17.37)	0.578
*Outcome of admission*			
Discharge	18 (17.8)	83 (82.2)	
Death	32 (41.0)	46 (59.0)	**0.001**
*Clinical symptoms*			
Ascites			0.201
Mild	1 (16.7)	35 (83)	
Moderate	20 (38.5)	32 (61.5)	
Severe	23 (25.6)	67 (74.4)	
No ascites	6 (19.4)	25 (80.6)	
Fever	12 (37.5)	20 (62.5)	0.183
Infections	30 (42.8)	40 (57.2)	**0.038**
Pedal oedema	27 (27.8)	70 (72.2)	0.975
Jaundice	28 (35.9)	50 (64.1)	0.058
Chills	9 (45)	11 (55)	0.071
Abdominal pain	18 (28.1)	46 (71.9)	0.966
Weight loss	39 (27.3)	104 (72.7)	0.695
Encephalopathy	27 (47.4)	30 (52.6)	**<0.001**
UGI bleeding	6 (25)	18 (75)	0.731
Others	45 (29.6)	107 (70.4)	0.237

UGI: upper gastrointestinal; BP: blood pressure.

**Table 2:** Clinical characteristics of cirrhotic patients with AKI associated with and without ACLF.

Variable	AKI with ACLF(N = 16)	AKI without ACLF(N = 34)	*p* value
*Causes*			0.415
Alcohol	10 (62.4)	14 (41.2)	
Alcohol/HBV	0 (0)	1 (2.9)	
Alcohol/HBV/HCV	1 (6.3)	0 (0)	
HBV	4 (25.0)	13 (38.2)	
HCV	1 (6.3)	2 (5.9)	
NAFLD	0 (0)	1 (2.9)	
Unknown	0 (0)	3 (8.8)	
*Precipitating factors*			**0.012**
Ascites	0 (0)	8 (23.5)	
Gastroenteritis	0 (0)	3 (8.8)	
Infection	13 (81.3)	19 (55.8)	
NIL	0 (0)	2 (5.9)	
UGIB	3 (18.7)	2 (5.9)	
*Outcome*			**0.001**
Dead	16 (100%)	16 (47.1)	
Live	0 (0%)	18 (52.9)	
*Sex of patient*			0.71
Female	7 (43.8)	13 (38.2)	
Male	9 (56.2)	21 (61.8)	
*Duration of stay (days)*			0.305
Median (minimum, maximum)	6 (2, 11)	11.9 (2, 44)	

HBV: hepatitis B virus; HCV: hepatitis C virus; NAFLD: nonalcoholic fatty liver disease.

**Table 3:** Child-Pugh classification.

Child-Pugh class	Frequency	Percentage
Class A	16	8.9
Class B	47	26.3
Class C	116	64.8
Total	179	100.0

**Table 4:** Causes of liver cirrhosis.

Causes	Frequency	Percent
Alcohol	72	40.2
HBV	65	36.3
HCV	6	3.4
NAFLDX	5	2.8
Schistosomiasis	4	2.2
Alcohol/HBV/HCV	1	0.6
HBV/alcohol	8	4.5
HBV/HCV	2	1.1
HCV/alcohol	2	1.1
Alcohol/HBV/HCV	1	0.6
Unknown	13	7.3
Total	179	100

HBV: hepatitis B virus; HCV: hepatitis C virus; NAFLD: nonalcoholic fatty liver disease.

**Table 5:** Precipitating factors for all AKI.

	Frequency	Percent
Infection	30	60.0
Refractory ascites	8	16.0
Hypovolemia		
*UGIB*	*5*	*10.0*
*Gastroenteritis*	*5*	*10.0*
Unknown precipitant	2	4.0
Total	50	100

UGIB: upper gastrointestinal bleeding.

**Table 6:** Logistic regression analysis of AKI stage and its effect on in-hospital mortality.

Outcomes	Odds ratio	SE	*p* value	95% conf interval		Sig
Stage 1a	1	.	.	.	.	
Stage 1b	6	8.124	.186	.422	85.248	
Stage 2	10.286	12.139	.048	1.018	103.948	^∗∗^
Stage 3	48	63.119	.003	3.647	631.76	^∗∗∗^
Constant	.167	.18	.097	.02	1.384	^∗^

^∗∗∗^ *p* < .01, ^∗∗^*p* < .05, ^∗^*p* < .1.

**Table 7:** Laboratory parameters of the study participants.

Laboratory parameters	AKI, present (*N* = 50)	AKI, absent (*N* = 129)	*p* value
WBC (10^9^/l)	12.8044 (1.7, 23.9)	12.1487 (-26.8, 51)	0.907
Platelet count (10^9^/l)	154.58 (57.95, 251.21)	171.0698 (41.45, 300.69)	0.417
TOT. BILI (umol/l)	159.9896 (-16.49, 336.47)	84.5649 (-27.15, 196.71)	**0.001**
DIR. BILI (umol/l)	94.79 (-7.74, 197.32)	53.0938 (-24.37, 130.55)	**0.004**
Total protein (g/l)	67.582 (52.79, 82.37)	69.748 (53.93, 85.57)	0.404
Albumin (g/l)	25.186 (17.7, 32.68)	29.288 (21.41, 37.17)	**0.002**
ALT (U/l)	65.054 (-1.74, 131.84)	64.684 (21.07, 108.29)	0.965
AST (U/l)	103.5 (23.08, 183.92)	125.727 (14.74, 236.72)	0.209
ALP (U/l)	287.149 (77.53, 496.77)	457.904 (20.18, 895.62)	**0.016**
GGT (U/l)	248.205 (-32.79, 529.21)	270.728 (7.79, 533.67)	0.639
INR	2.942 (1.65, 4.23)	2.23 (1.45, 3.01)	**<0.001**
CPS	2.74 (2.18, 3.31)	2.48 (1.81, 3.15)	**0.017**
MELDNa	33.9 (26.71, 41.09)	22.11 (15.94, 28.26)	**<0.001**
Sodium (mmol/l)	130.214 (121.99, 138.43)	133.704 (128.03, 139.37)	**0.001**
Potassium (mmol/l)	4.331 (3.23, 5.43)	3.9506 (3.35, 4.650)	**0.005**
Creatinine (umol/l)	271.3548 (127.06, 415.74)	73.6643 (48.76, 98.64)	**<0.001**
BUN (umol/l)	17.6812 (5.1, 30.3)	5.4277 (2.24, 8.62)	**<0.001**

Abbreviations: ALT: alanine aminotransferase; ALP: alkaline phosphatase; GGT: gamma glutamyl transferase; AST: aspartate aminotransferase; BUN: blood urea nitrogen; WBC: white blood cell; CPS: Child-Pugh score; MELDNa: model for end-stage liver disease sodium; Cr: Creatinine; T. Bil.: total bilirubin; D. Bil.: direct bilirubin; ^∗^*p* < 0.05: statistically significant.

**Table 8:** Multivariable regression analysis of independent variables associated with AKI.

Variables	*B*	S.E.	Wald	*p* value	Odds ratio	95% C.I.	
TOT. BILI	-0.026	0.015	2.941	0.086	0.974	0.945	1.004
DIR. BILI	0.031	0.022	1.949	0.163	1.032	0.987	1.078
Albumin	0.059	0.059	0.973	0.324	0.943	0.839	1.060
ALP	-0.004	0.002	4.321	**0.038**	0.996	0.993	1.000
INR	-1.160	0.567	4.192	**0.041**	0.314	0.103	0.952
CPS	-0.462	0.240	3.696	0.055	0. 630	0.393	1.009
MELDNA	0.595	0.134	19.755	**<0.001**	1.813	1.013	2.357
Sodium	0.142	0.066	4. 683	**0.030**	1.153	1.019	1.311
Potassium	-0.366	0.512	0.510	0.475	0.694	0.254	1.893
BUN	0.210	0.080	6.902	**0.009**	1.234	1.055	1.443
Infection	1.524	0.866	3.097	0.078	4.589	0.841	2.043
ENCEP	-0.481	0.809	0.353	0.552	0.618	0.127	3.020
Constant	-28.238	10.383	7.396	0.007	0.000		

Abbreviations: ALP: alkaline phosphatase; BUN: blood urea nitrogen; CPS: Child-Pugh score; MELDNa: model for end-stage liver disease sodium; T. Bil.: total bilirubin; D. Bil.: direct bilirubin; ENCEP: encephalopathy; ^∗^*p* < 0.05: statistically significant.

## Data Availability

The data used to support the findings of this study are available from the corresponding author upon request.
